The article "Application of the Artificial Neural Network in the Diagnosis of Infantile Bronchial Bridge with 64-Slice Multislice Spiral CT" was retracted in 2023. Reasons: signs of a paper mill; suspected computer-generated content; unreliable results or conclusions; lack of ethics approval or compliance.

# Application of the Artificial Neural Network in the Diagnosis of Infantile Bronchial Bridge with 64-Slice Multislice Spiral CT

**DOI:** 10.1155/2021/3694664

**Published:** 2021-09-29

**Authors:** Gengwu Li, Chang Wang, Huihui Lin, Xu Li, Jun Hu

**Affiliations:** Department of Image, Anhui Provincial Children's Hospital, Children's Hospital of Fudan University in Anhui, Hefei 230051, China

## Abstract

The objective is to study the application of spiral CT in the diagnosis of the trachea in children. In this study, the effect of 64-slice multislice spiral CT in diagnosing infant bronchial bridge was studied based on an artificial neural network. From June 2020 to December 2020, 100 cases of children with the trachea in the outpatient department of our hospital were selected as the research object. They were divided into the study group and the control group, with 50 cases in each group. The results showed that among the 50 cases in the control group, 42 cases were found to have a bronchial foreign body and 8 cases were missed; the detection rate was 84%. There were 7 cases of trachea foreign body, 15 cases of left bronchial foreign body, 14 cases of right bronchial foreign body, and 6 cases of medium bronchial foreign body. The detection rate of the study group was significantly higher than that of the control group, with a statistical significance (*P* < 0.05). *Conclusion*. The detection rate of neural networks in MSCT is higher than that of X-ray, and the MSCT based on the artificial neural network can clearly show the morphology, position, and the relationship between the foreign body and trachea, which is worthy of clinical promotion and application.

## 1. Introduction

A bronchial foreign body is the most common accident in children, second only to car accidents, poisoning, and ranked the third accidental injury. If not timely diagnosis and treatment, it often endangers the life of children. Ordinary X-ray examination can only be diagnosed by indirect signs, not direct signs. However, when the obstruction signs are not obvious, an X-ray examination is easy to miss the diagnosis. Due to its isotropic characteristics, multislice spiral CT (MSCT) can directly display foreign bodies in the transverse position, the location and size of foreign bodies through three-dimensional reconstruction, providing a fast, accurate, and noninvasive examination method [1].

An artificial neural network (ANN) is a kind of information analysis and processing system based on imitating the structure and function of the human nervous system. It is a nonlinear mapping and adaptive dynamical system which is composed of a large number of simple neurons interconnected widely. ANN's inherent parallel structure, high fault tolerance, self-adaptability, and nonlinear comprehensive reasoning ability provide a new and effective approach for diagnosing diseases. At present, the ANN has been widely used to diagnose chest diseases, including pulmonary embolism, interstitial pulmonary diseases, lung cancer, and breast lesions. However, it is rarely used in imaging the diagnosis of abdominal diseases.

The article "Application of the Artificial Neural Network in the Diagnosis of Infantile Bronchial Bridge with 64-Slice Multislice Spiral CT" was retracted in 2023. Reasons: signs of a paper mill; suspected computer-generated content; unreliable results or conclusions; lack of ethics approval or compliance.

Infant tracheal and bronchial foreign body is one of the common emergencies in paediatrics and otolaryngology department. The onset is usually relatively urgent. The children appear with wheezing, dyspnea, purple, asphyxia, other clinical symptoms, and even life-threatening in severe cases. Because the child is young, it is often unable to accurately express and provide the medical history, which is prone to missed diagnosis and misdiagnosis. Clinicians need to routinely conduct relevant examinations after receiving the treatment to help further diagnosis treatment. How to obtain clinically satisfactory and diagnostic images while reducing the dose is the goal of our research. Through retrospective analysis of some cases in our hospital in recent two years, the image quality and radiation dose are obtained under different scanning machines and different scanning modes to further explore the clinical value of Xikouzi dual-source Flash scan in the diagnosis of infant bronchial foreign body [2]. Children are under five years of age due to the imperfect development of many functions such as chewing and laryngeal reflex. If they cry, laugh, slap, and play, while eating, foreign objects are easily inhaled into the trachea, causing irritating cough, shortness of breath, anxiety, wheezing, and delicate complexion. When the foreign body is small, the clinical symptoms are mild, sometimes accompanied by breathing movement to change the position of the foreign body. Obstructive emphysema often occurs when the exhalation valve is blocked because the lung lobe where the lesion is located cannot be discharged normally. When inhalation valve obstruction occurs, the external oxygen cannot be supplied to the distal end of the lung lobes. It is easy to cause lung atrophy, obstructive pneumonia, or atelectasis due to hypoxia. Larger bronchial foreign bodies can usually directly cause obstructive pneumonia or atelectasis. In severe cases, the condition is dangerous, and suffocation and death are even possible [3]. Prompt and correct diagnosis and treatment can reduce the risk of asphyxia or other complications in children. Doctors can take effective treatment measures in time, which is very important to reduce mortality. For patients with any foreign body in the hypochondria, general primary hospitals routinely use X-ray examination first, including fluoroscopy, CR, or D civilian film examination. There are many kinds of foreign bodies. On clinical imaging, foreign bodies are often divided into positive opaque foreign bodies and negative transparent foreign bodies. If it is a positive foreign body, such as coins, screws, keys, metal buttons, or batteries, it is easy to find the foreign body under the X line. Doctors will determine the location of the foreign body according to intuitive judgment, and the foreign body can be removed directly by tracheoscopic surgery. If the foreign body is negative, X-ray examination often has large limitations. Eight can only be determined by some indirect signs, including emphysema, pulmonary inflammatory lesions, mediastinal swing, and other signs. Mild emphysema is often difficult to be found in ordinary X-ray examinations [4]. According to some data, X-ray diagnosis of bronchial foreign body diagnostic coincidence rate is about 40–50%, but its low price, convenient operation, is still one of the screening methods commonly used in primary hospitals. Chest fluoroscopy can be used to observe the patient from multiple angles and directions. It can be more convenient to observe some pulmonary complications, thus helping to determine whether there is a possibility of airway foreign bodies. X-rays alone have a diagnostic rate of about 50%. Chest X-rays have a higher diagnostic accuracy of 89% than conventional X-rays. CT has been developed rapidly in recent years. The scanning equipment routinely is used in our hospital including 64-slice spiral CT, second-generation new dual-source; 64-slice CT is single-emission CT. It is also a conventional examination device used in the emergency department of our hospital. It has the advantages of fast scanning speed and high image resolution. Dual-source CT is a relatively new device; dual-source CT has two spherical tubes that integrate two sets of 64-layer X-ray emission sources and two detectors into a single machine. This design idea has many technical advantages that single-source CT is not prepared for, and it is a milestone breakthrough in the history of CT development [5]. Ma et al. proposed diagnosing the artificial neural network-assisted CT image in medicine [6]. Mohandes et al. showed that CT has high sensitivity and specificity in the imaging diagnosis of the trachea and bronchial foreign bodies, with an accuracy of up to 97%, providing outstanding contributions to the diagnosis and differential diagnosis of difficult cases [7]. Binek et al. showed that dual-source CT, with its new hardware and software technology advantages and powerful postprocessing function, is very suitable for examining suspected bronchial foreign bodies in children [8]. A total of 100 children with trachea treated in the outpatient department of our hospital from June 2020 to December 2020 were selected as the research objects by an artificial neural network. They were divided into the study group and control group, with 50 cases in each group. The results showed that foreign bodies in bronchial tubes in the control group were detected in 42 cases and missed diagnosis in 8 cases, with a detection rate of 84%. There were seven tracheal foreign bodies, 15 left bronchial foreign bodies, 14 right bronchial foreign bodies, and 6 middle bronchial foreign bodies. The detection rate in the study group was significantly higher than that in the control group, and the difference was statistically significant (*P* < 0.05). The detection rate of MSCT is higher than that of X-ray, and MSCT can clearly show the morphology, location, and relationship between foreign body and trachea, which is worthy of clinical promotion and application.

The article "Application of the Artificial Neural Network in the Diagnosis of Infantile Bronchial Bridge with 64-Slice Multislice Spiral CT" was retracted in 2023. Reasons: signs of a paper mill; suspected computer-generated content; unreliable results or conclusions; lack of ethics approval or compliance.

## 2. Research Methods

### 2.1. Clinical Data

A total of 100 children with tracheal and bronchial foreign bodies who visited the outpatient department of our hospital from June 2020 to December 2020 were selected as the research objects. All the children were randomly divided into the study group and control group, with 50 cases in each group, including 70 males and 30 females, The age ranged from 7 months to 11 years and five months, the mean age was (74.12 ± 3.15) months, the course of the disease was 1 hour to 12 days, and the mean course of the disease was 4.23 ± 2.48 days. The clinical manifestations of the children are irritant cough, varying degrees of dyspnea, cyanosis, and other symptoms, and some of the children also have fever, shortness of breath, or asthma. Sixty-five patients had a clear history of foreign body inhalation, and 35 patients had no apparent history of foreign body inhalation. All children were confirmed by fiberoptic bronchoscopy or clinical diagnosis. There were no significant differences between the two groups in age, gender, disease, and medical history (*P* > 0.05), indicating that the two groups were comparable.

### 2.2. Establishment and Training of the Neural Network Model

This study adopts the error backpropagation (BP) neural network, which is widely used and mature at present. The network consists of two layers. The neural network structure is as follows: 14 input variables, 7 neurons in the hidden layer, and 1 neuron in the output layer, and the transfer function of the neurons in the hidden layer and output layer is logsig function (Figure 1). One hundred clinical children with trachea and bronchial foreign bodies were collected from June 2020 to December 2020. The train function is used to train the generated neural network. To improve the generalization ability of the network, that is, the network's ability to process new input samples, training is carried out in combination with the “early stopping method.”

The article "Application of the Artificial Neural Network in the Diagnosis of Infantile Bronchial Bridge with 64-Slice Multislice Spiral CT" was retracted in 2023. Reasons: signs of a paper mill; suspected computer-generated content; unreliable results or conclusions; lack of ethics approval or compliance.

### 2.3. Observation Indicators

The location, shape, size, and degree of obstruction of foreign bodies in the trachea and bronchus were observed and recorded. MSCT was compared with conventional X-ray examination and microscopic examination.

### 2.4. Statistical Methods

Statistical processing was performed on the obtained data, and SPSS15.0 software was used for analysis. The measurement data were analyzed by the *t*-test, and the enumeration data were analyzed by the *χ*^2^ test. *P* < 0.05 was considered statistically significant.

## 3. Research Results

### 3.1. Results of MSCT

In the study group, foreign bodies in bronchial tubes were detected in 38 cases and missed diagnosis in 12 cases, with a detection rate of 76%. There were 9 cases of tracheal foreign body, 16 left bronchi, 9 cases of right bronchus, and 4 cases of the middle bronchus.

### 3.2. Network Training Results after the Training Program Runs

The above training process shows that after the 12th step of training, the verification error starts to increase, and the training stops. It can be seen that the variation trend of verification error and testing error is basically the same, which indicates that the sample set partition is reasonable in training. The two training error curves show that the neural network converges quickly and the convergence error is small in the training process, and the training effect of the network is good (Figure 2).

### 3.3. Comparison of the Results of the Two Examination Methods

Based on the artificial neural network MSCT and abstract MSCT to detect foreign bodies in the trachea and bronchus of children, the detection rates of the study group and the control group were 84% and 76%, respectively. Comparing the results of the two groups, the detection rate of the study group was significantly higher than that of the control group. The difference was statistically significant (*P* < 0.05), as given in Table 1.

### 3.4. Species of Foreign Bodies

Bronchial foreign bodies were detected in 93 of the 100 children, including 84 cases of plantlike foreign bodies, including peanuts, sunflower seed skins, corn kernels, watermelon seeds, and nuts. There were 8 cases of nonplant foreign bodies, including metal buckles, whistles, plastic pen caps, plastic toys, chicken bones, and fish bones.

The article "Application of the Artificial Neural Network in the Diagnosis of Infantile Bronchial Bridge with 64-Slice Multislice Spiral CT" was retracted in 2023. Reasons: signs of a paper mill; suspected computer-generated content; unreliable results or conclusions; lack of ethics approval or compliance.

The favourable rates of MSCT, chest fluoroscopy, and X-ray were 100%, 88.89%, and 48.83%, respectively. Among the imaging examinations of suspected bronchial foreign body, MSCT had the highest accuracy, and chest fluoroscopy is inferior to chest X-ray. The mutual night was statistically significant (*P* < 0.01), as given in Table 2.

The artificial neural network-assisted diagnosis model established in this study is based on the extraction of multislice spiral CT imaging features. This process is completed by radiologists' analysis and interpretation. It is greatly influenced by subjective factors, and the diagnostic results are closely related to the medical level of doctors. Then, on how to intelligently extract the features of multilayer CT images for further research, establish an artificial intelligence network intelligent diagnosis model for infant bronchial CT images, eliminate various human factors throughout the diagnosis process, and obtain a more comprehensive, accurate, and objective diagnosis. Improve the correct diagnosis rate of infant bronchus, especially early infant bronchus, so that more patients can receive timely and effective treatment.

## 4. Results and Discussion

The objective is to explore the application of spiral CT in trachea diagnosis in children. An artificial neural network-based 64-slice spiral CT method in infant bronchial bridge diagnosis is presented. A total of 100 children with trachea in the outpatient department of our hospital from June 2020 to December 2020 were selected as the research objects and divided into the study group and the control group, with 50 cases in each group. The results showed that among the 50 cases in the control group, 42 cases were detected and 8 cases were missed. The detection rate was 84%. There were 7 cases of trachea foreign body, 15 cases of left bronchial foreign body, 14 cases of right bronchial foreign body, and 6 cases of medium bronchial foreign body. The detection rate of the study group was significantly higher than that of the control group. The difference was statistically significant (*P* > 0.05). It is proved that multislice spiral CT based on an artificial neural network can clearly display the morphology, position, and the relationship with trachea of foreign bodies, which is worthy of clinical application. Specifically reflected in the establishment of the artificial network of the infant bronchial CT image intelligent diagnosis model, the entire diagnosis process is to eliminate all kinds of human factors, more comprehensive, accurate, and objective diagnosis, and improve the infant bronchial, especially early infant bronchial correct diagnosis rate, so that more patients get timely and effective treatment.

The article "Application of the Artificial Neural Network in the Diagnosis of Infantile Bronchial Bridge with 64-Slice Multislice Spiral CT" was retracted in 2023. Reasons: signs of a paper mill; suspected computer-generated content; unreliable results or conclusions; lack of ethics approval or compliance.

## Figures and Tables

**Figure 1:** Schematic diagram of the neural network object structure.

**Figure 2:** Network training process.

**Table 1:** Comparison of results of the two inspection methods.

Group	The number of cases	Confirmed	Detection rate (%)
The team	50	42	84
The control group	50	38	76

**Table 2:** Comparison of accuracy of three different imaging methods for the bronchial foreign body.

	Chest X-ray, A	Chest fluoroscopy, B	MSCTC
Positive	9	27	14
Negative	12	3	0
A combined	21	30	14

## Data Availability

The data used to support the findings of this study are available from the corresponding author upon request.
